# Development of a 5-Gene Signature to Evaluate Lung Adenocarcinoma Prognosis Based on the Features of Cancer Stem Cells

This article has been retracted.

**DOI:** 10.1155/2022/4404406

**Published:** 2022-04-16

**Authors:** Renping Wan, Hongliang Liao, Jingting Liu, Lin Zhou, Yingqiu Yin, Tianhao Mu, Jie Wei

**Affiliations:** ^1^Department of Thoracic Surgery, Yuebei People's Hospital, 133 Huimin South Road, Wujiang District, Shaoguan City, Guangdong Province, China 440200; ^2^Department of Respiratory Medicine, Yuebei People's Hospital, 133 Huimin South Road, Wujiang District, Shaoguan City Guangdong Province, China 440200; ^3^Department of Oncology, HaploX Biotechnology, 8/F, Aotexin Power Building, No. 1, Songpingshan Road, High Tech North District, Nanshan District, Shenzhen City, Guangdong Province, China 440300; ^4^Department of Biomedical and Health Engineering, Shenzhen Institute of Advanced Technology, Chinese Academy of Sciences, 1068 Xueyuan Avenue University Town, Nanshan District, Shenzhen City, Guangdong Province, China 440300

## Abstract

Cancer stem cells (CSCs) can induce recurrence and chemotherapy resistance of lung adenocarcinoma (LUAD). Reliable markers identified based on CSC characteristic of LUAD may improve patients' chemotherapy response and prognosis. OCLR was used to calculate mRNA expression-based stemness index (mRNAsi) of LUAD patients' data in TCGA. Association analysis of mRNAsi was performed with clinical features, somatic mutation, and tumor immunity. A prognostic prediction model was established with LASSO Cox regression. Kaplan-Meier Plotter (KM-plotter) and time-dependent ROC were applied to assess signature performance. For LUAD, univariate and multivariate Cox analysis was performed to identify independent prognostic factors. LUAD tissues showed a noticeably higher mRNAsi in than nontumor tissues, and it showed significant differences in T, N, M, AJCC stages, and smoking history. The most frequently mutated gene was TP53, with a higher mRNAsi relating to more frequent mutation of TP53. The mRNAsi was significantly negatively correlated with immune score, stromal score, and ESTIMATE score in LUAD. The blue module was associated with mRNAsi. The 5-gene signature was confirmed as an independent indicator of LUAD prognosis that could promote personalized treatment of LUAD and accurately predict overall survival (OS) of LUAD patients.

## 1. Introduction

Lung adenocarcinoma (LUAD) originates from small airway epithelial type II alveolar cells [1, 2]. Most LUAD patients are diagnosed at advanced cancer stages; conventional treatments for those patients are chemotherapy and radiation, to which LUAD is highly resistant. Thus, LUAD shows a high mortality, the five-year survival chance of which is about 15% [3, 4]. This also demands better improvement of early diagnosis, survival prediction, and relapse monitoring of LUAD patients to prolong their survival.

A study found cancer stem cells (CSCs) as a small subgroup of cancer cells with stemness. The self-renewing of CSCs and their production of differentiated cells could facilitate the formation of tumor heterogeneity [5]. The latest evidence indicated that CSC-mediated stem-like phenotypes of cancer cells are the major factor responsible for cancer recurrence and chemical resistance [6]. This also points to the need to accurately identify CSC population. However, due to the quiescent nature of lung epithelial cells, distinguishing normal lung epithelial cells from lung CSCs is still a great challenge [7]. A study showed that identifying CSC markers may help characterize CSCs [8]. In LUAD, several CSC markers, including CD44 [9], CD90 [10], and SOX2, have been discovered [11], but clinical application of CSC-specific biomarkers is less popular. Furthermore, the fact that most markers could mark heterogeneous stem cell populations suggests that their isolation and characterization should be developed using a combination of surface markers or a combination of intracellular or extracellular markers [12]. Malta et al. [13] developed a new indicator to reflect stem cell features of mRNAsi calculated by OCLR. Their results proved that a higher value of mRNAsi is indicative of stronger characteristics of CSCs.

At present, there are several system biology methods to identify biomarkers related to the prognosis of LUAD and construct mRNA features. Li et al. [14] identified a 7-gene signature by a nonnegative matrix factorization (NMF) method using gene expression profile related to lipid metabolism, Shi et al. [15] established three TKI-related gene expression profiles to predict the chemosensitivity of lung cancer patients. Zhang et al. [16] identified seven gene markers to predict the prognosis of lung cancer patients by using multiomics data integration analysis. The authors of the three groups tested their gene signatures in internal and external data sets but did not conduct clinical verification. This means that identifying robust gene signatures is still a challenge, and more queues are needed to verify signatures. In conclusion, it is very important to identify the gene characteristics related to the prognosis of LUAD by bioinformatics analysis of its biological function. In this study, clinical LUAD data were derived from TCGA database, and mRNAsi was calculated based on OCLR to investigate the relationship of mRNAsi and clinical LUA characteristics and mutations of LUAD. The weighted gene coexpression network analysis (WGCNA) was constructed for screening modules associated with mRNAsi, according to which genes showing a significance of prognostic relevance to LUAD were filtered. Finally, a 5-gene independent prognostic signature was established that may be beneficial for optimizing survival risk assessment and personalized management of patients with LUAD.

## 2. Materials and Methods

### 2.1. Data Acquisition and Research Design

From the PCBC website, RNA-Seq data for pluripotent stem cell samples were acquired using the R package synapser (v 0.6.61). The data of induced pluripotent stem cells (IPSC) samples and embryonic stem cell (ESC) were retained. The Ensembl IDs of ESC and IPSC samples were reserved and converted into gene symbol to retain only protein-encoding genes. The data of 78 samples were obtained. From TCGA database, clinical LUAD data containing RNA-Seq profilation information of 594 samples were acquired. The microarray GSE31210 (*n* = 246) and GSE50081 (*n* = 181) were downloaded from GEO website (Table S1). Each LUAD sample had expression profile information and survival data. The median expression value of multiple gene symbols was taken, whereas probes corresponding to multiple genes were excluded. The comprehensive gene annotation is obtained from the GENCODE database (GRCh38.p13), and the information is used to map the Ensembl ID to the gene symbol, and only the protein-encoding genes were reserved.  Figure 1 summarizes our study design.

### 2.2. Correlation between mRNAsi and Clinical Features

mRNAsi was calculated according to the OCLR method provided by Malta et al. [13]. mRNAsi differences between tumor samples and normal samples were analyzed by an unpaired *t*-test. We used one-way ANOVA in mRNAsi difference comparison between groups of patients in terms of gender, age, clinical stage, TNM stage, and smoking history.

### 2.3. Relational Analysis between mRNAsi and Molecular Subtypes

MuTect [17] detection on TCGA-LUAD was performed using TCGAbiolinks [18] (V2.14.0), and differences in mRNAsi of different molecular mutant subtypes were analyzed. In addition, molecular subtype of TCGA-LUAD samples was also extracted using R package TCGA biolinks. mRNAsi differences between samples classified by the CIMP or iCluster were compared.

### 2.4. Weighted Gene Coexpression Network Analysis (WGCNA)

For constructing a coexpression network [19], the WGCNA algorithm was performed. After removing outlier samples, Pearson's correlation coefficients were determined between groups of genes. The optimal efficacy value *β* was chosen to construct proximity matrix, which was transformed into topological overlap matrix (TOM). For gene cluster according to TOM (in each gene network module, the minimum number of genes was 80), an average-linkage hierarchical clustering method was applied. The pruning algorithm was applied to divide gene modules and integrate those close modules. The most relevant modules with mRNAsi were screened by correlation analysis.

### 2.5. Functional Enrichment Analysis

The R software (https://www.R-project.org/,version 4.0.2) packageWebGestaltR [20] (v0.4.2) was employed to perform KEGG and GO functional enrichment analyses for analyzing potential biological functions of the most relevant modules of mRNAsi obtained from WGCNA. GO categories were cellular component (CC), molecular function (MF), and biological process (BP). A statistical significance was defined when FDR < 0.05 and *P* < 0.05.

### 2.6. Construction and Verification of Prognostic Signature

Genes of mRNAsi-related modules were separated into verification and training sets based on the principle of the same sample size (Table 1). To analyze the relevance between genes and OS (statistical significance was *P* < 0.01), Univariate Cox analysis was used here. Glmnet software (doi:10.18637/jss.v039.i05, version 4.1-2) package was used for LASSO Cox regression analysis. Here, those genes of a *P* < 0.05 were further refined according to the Akaike Information Criterion (AIC). The risk score was determined for each patient by multiplying risk factor obtained by Lasso Cox with gene expression extracted. After standardization, with 0 as the threshold, the samples were grouped by the risk scores into two risk groups (low and high). For OS comparisons between risk groups, we plotted Kaplan-Meier (KM) survival curve. ROC curves were used for prediction evaluation of the signature. In addition, previous LUAD prognostic models were compared with the current risk model.

### 2.7. The Construction of a Nomogram

To precisely determine independent LUAD prognostic factors, clinical parameters, including gender, age, AJCC stage, T stage, and risk score were subjected to univariate and multivariate Cox regression analyses. Using these clinical factors, a nomogram for OS analysis in 1, 3, and 5 year(s) was built.

## 3. Results

### 3.1. mRNAsi and Clinical Characteristics of LUAD

See Figure 1 for the work flow of the current work. mRNAsi, which is a new stemness index for dedifferentiation potential evaluation of tumor cells, has been regarded as a CSC marker [21]. mRNAsi was noticeably higher in LUAD tissues than nontumor ones (Figure 2(a)). The clinical features of mRNAsi in LUAD were examined. The divisions of LUAD patients were divided into two groups according to gender, and age showed no significant difference in mRNAsi between age > 65 and age ≤ 65 (Figure 2(c)), but mRNAsi significant differences in N stage (Figure 2(e)), gender (Figure 2(b)), AJCC stage (Figure 2(g)), and smoking (Figure 2(h)), T stage (Figure 2(d)), and M stage (Figure 2(f)) were observed. Hence, mRNAsi was associated with TNM stage, AJCC stage, and smoking.

### 3.2. Associations of mRNAsi with Mutations

The somatic mutation spectrum of LUAD patients was analyzed by maftools.  Figure 3(a) shows the top 10 most frequently genes (KRAS, TTN, TP53, MU16, ZFHX4, Ush2a, CSMD3, LRP1b, RyR2, and XIRP2); here, the gene showing the most frequent mutation was TP53. The mRNAsi differences of each gene between the mutated and nonmutated samples were further analyzed, and the mRNAsi of TTN-, LRP1B-, TP53-, CSMD3-, ZFHX4-, MU16-, USH2A-, XIRP2-, and RyR2-mutated samples were greatly higher than that of nonmutated samples (Figures 3(b)–3(j))3. To further examine the relationship between mRNAsi of tumor samples and clinical features and molecular mutations, tumor samples were arranged according to mRNAsi from low to high, and the clinical data and mutation trends of different samples with mRNAsi were compared. The results demonstrated that the mortality and AJCC stage of patients were increased with the increase of mRNAsi. In addition, a higher mRNAsi was indicative of more frequent mutations of CSMD3, TTN, MU16, RyR2, and TP53 (Figure 4).

### 3.3. Correlation of mRNAsi with Molecular Subtypes and Tumor Immunity

To understand the mRNAsi differences between subtype groupings, LUAD samples were grouped according to CpG Island methylator phenotype (CIMP) or iCluster [22]. According to CIMP, the LUAD samples were divided into three subtypes, and significant differences in mRNAsi among the three subtypes were observed (Figure 5(a)). iCluster analysis detected six clusters in LUAD, with significant differences in mRNAsi among them (Figure 5(b)). We also investigated the association of mRNAsi with tumor immunity. ESTIMATE software (https://sourceforge.net/projects/estimateproject/) package was employing for immune and matrix score determination of LUAD samples, and Pearson's correlation analysis showed that in LUAD, ESTIMATE score, immune score, and stromal score were significantly negatively linked to mRNAsi (Figures 5(c)–5(e)), indicating that mRNAsi was involved in tumor immunity.

### 3.4. Filtering mRNAsi-Related Gene Modules and Their Functions

WGCNA developed the coexpression network for identifying mRNAsi-related modules. Correlation coefficient in this study was >0.85 when *β* = 6 (Figure 6(a)). Therefore, a soft threshold of 6 was employed to establish a scale-free network; here, we obtained 14 gene modules (Figure 6(b)). The correlation of each module to LUAD patients' age, T stage, gender, smoking, N stage, AJCC stage, M stage, mRNAsi was analyzed; here, the blue module is the most associated with mRNAsi (Figure 6(c)). The biological processes involved in the blue module were explored using Gene Ontology (GO) and Kyoto Encyclopedia of Genes and Genomes (KEGG). The blue module was found to be largely implicated in cell mitogen-related pathways, including organelle fission, ribonucleoprotein complex biogenesis, and ncRNA metabolic process (Figure 6(d)). From KEGG analysis, the blue module was mainly concentrated with DNA replication, homologous recombination, base excision repair, etc. (Figure 6(e)).

### 3.5. Construction of the 5-Gene Signature Based on mRNAsi-Related Genes

A total of 2297 genes were extracted from the blue module by univariate Cox analysis, and 268 survival-related genes in LUAD were retained (Table S2). Nine prognosis-associated genes for LUAD patients were identified with LASSO Cox. According to AIC, 4 genes were eliminated, while the remaining 5 genes were used to build prognostic signature: Risk score = 0.117∗PKP2 + 0.340∗GNPNAT1 + 0.299∗H2AFX + 0.263∗TLE1 + 0.459∗AVEN (Figure S1). TCGA training set samples were classified into two risk groups (low and high) through calculating each sample's risk score using the 5-gene signature (Figure 7(a)). Survival analysis revealed a better prognosis of low-risk LUAD patient group (Figure 7(b)). For 1-year, 3-year, and 5-year OS, the AUC of the risk score was 0.7, 0.76, and 0.65, respectively (Figure 7(c)).

### 3.6. Internal and External Verification of the 5-Gene Signature

To assess the prediction of the 5-gene signature, further validation was performed in four queues (TCGA validation set, complete TCGA-LUAD data set, GSE31210, and GSE50081). According to the risk score, cohort samples were categorized into two groups (low and high) (Figure 8(a)). We found that in TCGA validation set, complete TCGA-LUAD dataset, GSE31210, and GSE50081, prognosis of LUAD patients with a low risk was greatly better than high-risk ones with significant differences (Figure 8(b)). From the ROC analysis on the AUCs of long-term survival, we found that the 5-year survival was higher than 0.6 in the four cohorts (Figure 8(c)). These results confirmed that the 5-gene signature predicted LUAD survival accurately.

### 3.7. Independent Prediction of the 5-Gene Signature in LUAD Prognosis

We explored the relationship of risk score to clinical characteristics, such as M stage, gender, T stage, AJCC, age, N stage, and smoking. As shown in Figure 9, all of these clinical characteristics showed a close relation to the risk score. For verifying the effectiveness of 5-gene signature, stratified analysis was conducted on age (age > 65 and age ≤ 65), AJCC stage (stage III-IV, stage I-II), gender (male and female), M stage (N2-N3 and N0-N1), T stage (T3-T4, T1, and T2), and N stage (M0). The results verified an effective OS prediction of the risk model in almost all subgroups apart from N2-N3 stage patients (Figure 10). Next, a nomogram was established through combining gender, age, risk score, AJCC stage, and T stage. Here, the risk score showed the greatest impact on the prediction of OS (Figure S2A). Moreover, AJCC stage and risk score were independent prognostic factors for LUAD, as verified by the data from univariate and multivariate Cox analysis (Table 2).

### 3.8. The 5-Gene Signature Outperformed the Other Three Signatures in Predicting the Performance of the OS

We also compared the 5-gene signature with three previously developed signatures [23–29]. TCGA samples' risk score were, respectively, determined using the seven signatures, and accordingly, all patients were divided to two risk groups (low and high). The survival analysis revealed a significant prognosis difference in the two groups (Figures 11(a), 11(c), 11(e), 11,11,11,11). ROC curve of the seven signatures showed that the AUCs for the survival in 1, 3, and 5 year(s) were both lower than 0.75 and the average AUC of OS predicted by our 5-gene signature (Figures 11(b), 11(d)11(f), 11,11,11,11), which indicated a high accuracy and performance of our signature.

### 3.9. Functional Analysis and Immune Correlation Analysis of 5-Gene Signature

In order to clarify the potential regulatory mechanism of 5-gene signature, we used ssGSEA method to calculate the KEGG pathway enrichment score of each patient and further calculated the correlation between 5-gene signature and each pathway. We can observe the relationship between 5-gene signature and p53_SIGNALING_PATHWAY, MISMATCH_REPAIR, DNA_REPLICATION, and CELL_Cycle, and other pathways were significantly positively correlated with Fatty_ACID_METABOLISM and ARACHIDONIC_ACID_Metabolism, and other metabolic pathways were significantly negatively correlated (Figure S3A). In addition, we also observed a significant positive correlation between 5-gene signature and mRNAsi (Figure S3B) and a significant negative correlation between 5-gene signature and immune infiltration (Figure S3C-E). The five genes contained in 5-gene signature were significantly overexpressed in tumor samples (Figure S3F). We also analyzed the correlation between the expression of five genes contained in 5-gene signature and mRNAsi. It can be observed that except TLE1 gene, the other four genes showed significant positive correlation with mRNAsi (Figure S3J-K).

## 4. Discussion

Local and/or systemic treatment of LUAD has been greatly improved, but posttreatment recurrence is still relatively frequent [30]. The regrowth of such tumors after treatment is now thought to be dependent on a few CSCs [31]. Ongoing trials demonstrated that anti-CSC therapy can increase tumor response to chemotherapy and improve patient outcomes [8]. As CSCs consist of a variety of heterogeneous phenotypes rather than a single cell type, predicting the effectiveness of a specific therapy to target CSC could be difficult. Therefore, CSC-specific regulatory pathways or markers that are characteristic of LUAD should be developed along with anti-CSC therapies [32]. Here, we evaluated the CSC characteristics of LUAD samples based on mRNAsi and calculated mRNAsi for each sample in TCGA database using OCLR. Previous studies have shown that compared with normal tissue, mRNAsi is significantly higher in tumor tissues such as breast cancer tissue [33], gastric cancer tissue [34], liver cancer tissues [35], and lung squamous cell carcinoma [36]. At this point, the analytical data revealed a significantly lower mRNAsi in nontumor tissues than LUAD tissues and that mRNAsi showed great differences in M stage, N stage, smoking, AJCC stage, and T stage. Multiple studies demonstrated that LUAD had a high rate of somatic mutation and genome rearrangement [22]. In recent years, a number of somatic mutations occurring in LUAD, including TP53, KRAS, PIK3CA, and MET, have been discovered [37]. Our work found that TP53 was the gene with the highest mutation frequency in LUAD, which was also consistent with previous studies. It is reported that TP53 mutation had a negative impact on cancer prognosis and is associated with a shorter survival time [38]. The status of TTN mutation can be applied to independently evaluate immunotherapy prognosis of LUAD patients [39]. Loss of CSMD3 function resulted from somatic mutations can stimulate the oncogenic transformation of airway epithelial cells [40]. RYR2 has been considered a mutated driver of lung cancer [41]. Somatic mutations of LRP1B are linked to lung tumor mutation load [42]. Here, a higher mRNAsi was correlated with more frequent mutations of XIRP2, MU16, ZFHX4, CSMD3, TTN, USH2A, TP53, RyR2, and LRP1B, without significant mRNAsi difference in mutant KRAS or wild-type KRAS.

A study found that CSCs can shape immune microenvironment of tumors, and in turn, the functional and phenotypic characteristics of tumor-infiltrating immune cells could affect the phenotype and differentiation of tumor cells [43]. This study then explored the association of tumor immunity to mRNAsi and confirmed that mRNAsi was closely correlated with ESTIMATE score, immune score, and stromal score of LUAD. Then, WGCNA showed that blue module was found to have the strongest correlation with mRNAsi; moreover, the module was mainly involved in pathways related to cell division. The accumulation of cell division of stem cells will lead to cancer development [44].

Based on the blue module, we developed a 5-gene signature and verified its reliability and independence in four cohorts. Previous studies reported the role of five genes in LUAD. It has been found that high-expressed PKP2 could result in a poor LUAD prognosis. Functionally, PKP2 knockdown inhibits the invasion, proliferation of lung cancer cells *in vitro*, and xenograft lung tumor growth *in vivo* [45]. GNPNAT1 has been detected to be significantly higher in LUAD in comparison with normal ones and is linked to tumor size, lymphatic metastasis status, and clinical stage of the patients [46]. GNPNAT1 is associated with prognosis and immune infiltration in LUAD [47]. H2AFX, which is considered one of the key genes related to mRNAsi, is also associated with the prognosis and cell cycle of LUAD [48]. TLE1 is identified as a lung-specific oncogene that regulates the EMT of A549 cells through inhibiting E-cadherin [49]. Aven has critical functions in cancer cell response to radiation therapy [50]. However, heterogeneity of LUAD will reduce the reliability of a single gene than the use of a combination of multiple genes.

The present work performed a comprehensive study of LUAD patients based on mRNAsi, screened the blue modules most associated with mRNAsi by WGCNA, and developed 5-gene signature for OS prediction of LUAD. The 5-gene signature showed a higher AUC in short-term OS prediction in both validation and training sets but was much lower in long-term prediction, suggesting that 5-gene signature is more suitable for predicting short-term survival of LUAD. Another limitation of this study was that all our data came from TCGA database, which lacked comprehensiveness. Moreover, biological experiments (*in vitro* and *in vivo)* should be conducted for result verification and further exploration, which will be conducted in our future study with systematic biological studies.

## Figures and Tables

**Figure 1:** Flowchart of research design.

**Figure 2:** mRNAsi and clinical characteristics of LUAD. (a) mRNAsi differences between neoplastic and normal tissues. (b) Differences in mRNAsi between female and male LUAD patients. (c) mRNAsi difference in LUAD patients with ge > 65 and age ≤ 65. (d) mRNAsi differences between LUAD patients at different T stages. (e) mRNAsi differences between LUAD patients at different N stage. (f) mRNAsi analysis of M1 stage, M2 stage, and M3 stage patients. (g) mRNAsi differences among the four AJCC stage. (h) Differences in mRNAsi among grouped patients according to smoking.1 stands for life-long nonsmokers (fewer than 100 cigarettes during lifetime), 2 stands for current smokers (includes daily smokers and nondaily smokers or occasional smokers), 3 stands for current reformed smokers for >15 years, 4 stands for current reformed smokers for ≤15 years, and 5 stands for current reformed smokers; duration not specified = 5.

**Figure 3:** Associations of mRNAsi with mutations. (a) An overview of the mutant map in LUAD; only the 10 genes with the highest mutation frequency are shown here. (b) mRNAsi differences between TP53 mutant (MT) and TP53 wild-type (WT) samples. (c) Differences in mRNAsi between TTN mutant LUAD samples and TTN wild-type LUAD samples. (d) mRNAsi differences between MU16 mutant LUAD samples and MU16 wild-type LUAD samples. (e) mRNAsi difference in patients with CSMD3 mutant and CSMD3 wild-type. (f) mRNAsi was compared between RYR2 mutant LUAD and RYR2 wild-type LUAD patients. (g) mRNAsi in LUAD patients with mutant LRP1B was compared with that in LUAD patients without mutant LRP1B. (h) Difference analysis was used to compare the difference in mRNAsi between samples with and without mutations in USH2A. (i) Violin plots showed mRNAsi between LUAD samples with and without LRP1B mutations. (j) Differences between XIRP2 wild-type samples and XIRP2 mutant samples Violin diagram of mRNAsi.

**Figure 4:** Clinical data and mutation trends for LUAD samples with different mRNAsi.

**Figure 5:** Correlation of mRNAsi with molecular subtypes and tumor immunity. (a) mRNAsi differences between LUAD samples classified according to CIMP. (b) mRNAsi differences among molecular subtypes identified by iCluster. (c) Correlativity between mRNAsi and stromal score of LUAD samples in TCGA. (d) Pertinent analysis between mRNAsi and immune score of LUAD samples in TCGA. (e) Correlation analysis between mRNAsi and ESTIMATE score of LUAD samples in TCGA.

**Figure 6:** Identification of gene module associated with mRNAsi. (a) Analysis of network topology for various soft-thresholding powers. (b) Hierarchical clustering tree bases on the topological overlap dissimilarity. (c) Correlation between 14 gene modules and gender, age, T stage, N stage, M stage, AJCC stage, smoking, and mRNAsi. (d) Go analysis of the blue modules. (e) KEGG analysis of blue module.

**Figure 7:** Construction of 5-gene signature on account of mRNAsi-related genes. (a) In TCGA training set, distribution of the risk score, survival data, and the mRNA expression of prognosis signature. (b) Survival curves of LUAD patients in a TCGA training set. (c) ROC analysis for OS prediction in TCGA training set.

**Figure 8:** Internal and external verification of 5-gene signature. (a) Distribution of the risk score, survival data, and the mRNA expression of prognosis signature in different cohorts. (b) Survival curves of patients with LUAD in different cohorts in the high-risk and low-risk groups. (c) Time-dependent ROC analysis for OS prediction in four cohorts.

**Figure 9:** Correlation between risk score and each clinicopathologic feature. A *t*-test or one-way ANOVA determined the correlation between risk score and age (a), gender (b), T stage (c), N (d), M stage (e), AJCC stage (f), and smoking (g), respectively.

**Figure 10:** Kaplan-Meier stratification survival analyses in TCGA-LUAD data set, including age ≥ 65 (a), age ≤ 65 (b), male (c), female (d), T1 (e), T2 (f), T3-T4 (g), M0 (h), N0-N1 (i), N2-N3 (j), stage I-II (k), and stage III-IV (l).

**Figure 11:** Five-gene signature outperformed the other three signatures in predicting the performance of the OS. (a) Kaplan-Meier curve of prognosis in patients with TCGA-LUAD predicted by 8-gene signature. (b) ROC curve of the 8-gene signature for 1-, 3-, and 5-year OS. (c) Kaplan-Meier curve of prognosis in patients with TCGA-LUAD predicted by 3-gene signature. (d) ROC curve of the 3-gene signature for 1-, 3-, and 5-year OS. (e) Kaplan-Meier curve of 3-gene signature developed by Cheng Yue et al. for predicting prognosis of patients with TCGA-LUAD.(f) ROC curve of the 3-gene signature developed by Yue et al. for 1-, 3-, and 5-year OS. (g) Kaplan-Meier curve for predicting the OS of TCGA-LUAD patients based on the 6-gene risk model developed by Wang et al. (h) ROC curve analysis showing the prognostic prediction efficiency of the risk model. (i) Kaplan-Meier curve for predicting the OS of TCGA-LUAD patients based on the 7-gene risk model developed by Al-Dherasi et al. (j) ROC curve analysis showing the prognostic prediction efficiency of the 7-gene risk model.

**Table 1:** Data statistics of TCGA training set and validation set.

Clinical features	TCGA-train	TCGA-test	*P*
OS			
0	156	162	0.6421
1	94	88	
Gender			
Female	122	148	0.02488
Male	128	102	
T stage			
T1	82	85	0.1201
T2	143	124	
T3	17	28	
T4	8	10	
TX	0	3	
N stage			
N0	160	164	0.2326
N1	52	42	
N2	35	34	
N3	1	1	
NX	2	9	
M stage			
M0	165	167	0.4442
M1	15	9	
MX	70	74	
Stage			
I	131	137	0.8681
II	61	58	
III	39	41	
IV	15	10	
X	4	4	
Age			
≤65	111	126	0.3647
>65	133	120	
NA	6	4	

**Table 2:** Univariate and multivariate Cox analysis of all LUAD samples in TCGA dataset.

Variables	Univariable analysis				Multivariable analysis			
	HR	95% CI of HR		*P*	HR	95% CI of HR		*P*
		Lower	Upper			Lower	Upper	
Age	1.008	0.993	1.024	0.299	1.014	0.999	1.030	0.065
Gender	1.048	0.783	1.403	0.753	0.978	0.727	1.317	0.884
T stage	1.514	1.275	1.797	2.3*E* − 06	1.180	0.979	1.421	0.082
Stage	1.437	1.277	1.617	1.7*E* − 09	1.289	1.122	1.480	3.3*E* − 04
Risk score	1.739	1.509	2.004	2.2*E* − 14	1.737	1.489	2.025	2.0*E* − 12

## Data Availability

The datasets used in this study were openly available at GSE31210 (https://www.ncbi.nlm.nih.gov/geo/query/acc.cgi?acc=GSE31210) and GSE50081 (https://www.ncbi.nlm.nih.gov/geo/query/acc.cgi).

## Supplementary Materials

Supplementary 1 Figure S1: screening of genes associated with the prognosis of LUAD; A, B: Lasso Cox analysis. C: survival curves of LUAD samples with high and low expression of PKP2. D: GNPNAT1 expression was associated with LUAD survival. E: survival analysis of patients with high and low expression of H2AFX. F: survival analysis of patients with high and low expression of TLE1. G: Kaplan-Meier curves of patients with high and low expressed AVEN.

Supplementary 2 Figure S2: nomogram based on age, gender, T stage, and AJCC stage combined with risk score.

Supplementary 3 Figure S3: functional analysis and immune correlation analysis of 5-gene signature; A: KEGG pathway significantly related to 5-gene signature; B: scatter plot of correlation between 5-gene signature and mRNAsi; C-E: correlation between 5-gene signature and immune infiltration score; F: the expression and distribution of five genes in 5-gene signature were different between cancer and adjacent cancer; G-K: scatter plot of correlation between five genes in 5-gene signature and mRNAsi.

Supplementary 4 Table S1: clinical information of samples in different cohorts.

Supplementary 5 Table S2: univariate Cox analysis of 2297 genes.

## References

[1] Hutchinson B. D., Shroff G. S., Truong M. T., Ko J. P. (2019). Spectrum of lung adenocarcinoma. *Seminars in Ultrasound, CT, and MR*.

[2] Zappa C., Mousa S. A. (2016). Non-small cell lung cancer: current treatment and future advances. *Translational Lung Cancer Research*.

[3] Denisenko T. V., Budkevich I. N., Zhivotovsky B. (2018). Cell death-based treatment of lung adenocarcinoma. *Cell Death & Disease*.

[4] Spella M., Stathopoulos G. T. (2021). Immune resistance in lung adenocarcinoma. *Cancers*.

[5] Barbato L., Bocchetti M., Di Biase A., Regad T. (2019). Cancer stem cells and targeting strategies. *Cell*.

[6] Garcia-Mayea Y., Mir C., Masson F., Paciucci R., LLeonart M. E. (2020). Insights into new mechanisms and models of cancer stem cell multidrug resistance. *Seminars in Cancer Biology*.

[7] Shukla S., Khan S., Sinha S., Meeran S. M. (2018). Lung cancer stem cells: an epigenetic perspective. *Current Cancer Drug Targets*.

[8] Roy L., Cowden Dahl K. D. (2018). Can stemness and chemoresistance be therapeutically targeted via signaling pathways in ovarian cancer?. *Cancers*.

[9] Zhang C., Wang H., Wang X., Zhao C., Wang H. (2020). CD44, a marker of cancer stem cells, is positively correlated with PD-L1 expression and immune cells infiltration in lung adenocarcinoma. *Cancer Cell International*.

[10] Yan X., Luo H., Zhou X., Zhu B., Wang Y., Bian X. (2013). Identification of CD90 as a marker for lung cancer stem cells in A549 and H446 cell lines. *Oncology Reports*.

[11] Nakatsugawa M., Takahashi A., Hirohashi Y. (2011). SOX2 is overexpressed in stem-like cells of human lung adenocarcinoma and augments the tumorigenicity. *Laboratory Investigation*.

[12] Walcher L., Kistenmacher A. K., Suo H. (2020). Cancer stem cells-origins and biomarkers: perspectives for targeted personalized therapies. *Frontiers in Immunology*.

[13] Malta T. M., Sokolov A., Gentles A. J. (2018). Machine learning identifies stemness features associated with oncogenic dedifferentiation. *Cell*.

[14] Li T., Chen J., Liu J., Chen Q., Nie W., Xu M. D. (2022). A lipid metabolism-based seven-gene signature correlates with the clinical outcome of lung adenocarcinoma. *Journal of Oncology*.

[15] Shi Y., Xu Y., Xu Z. (2022). TKI resistant-based prognostic immune related gene signature in LUAD, in which FSCN1 contributes to tumor progression. *Cancer Letters*.

[16] Zhang S., Zeng X., Lin S., Liang M., Huang H. (2022). Identification of seven-gene marker to predict the survival of patients with lung adenocarcinoma using integrated multi-omics data analysis. *Journal of Clinical Laboratory Analysis*.

[17] do Valle I. F., Giampieri E., Simonetti G. (2016). Optimized pipeline of MuTect and GATK tools to improve the detection of somatic single nucleotide polymorphisms in whole-exome sequencing data. *BMC Bioinformatics*.

[18] Colaprico A., Silva T. C., Olsen C. (2016). TCGAbiolinks: an R/Bioconductor package for integrative analysis of TCGA data. *Nucleic Acids Research*.

[19] Langfelder P., Horvath S. (2008). WGCNA: an R package for weighted correlation network analysis. *BMC Bioinformatics*.

[20] Wang J., Vasaikar S., Shi Z., Greer M., Zhang B. (2017). WebGestalt 2017: a more comprehensive, powerful, flexible and interactive gene set enrichment analysis toolkit. *Nucleic Acids Research*.

[21] Pei J., Wang Y., Li Y. (2020). Identification of key genes controlling breast cancer stem cell characteristics via stemness indices analysis. *Journal of Translational Medicine*.

[22] (2014). Comprehensive molecular profiling of lung adenocarcinoma. *Nature*.

[23] Li S., Xuan Y., Gao B. (2018). Identification of an eight-gene prognostic signature for lung adenocarcinoma. *Cancer Management and Research*.

[24] Liu W. T., Wang Y., Zhang J. (2018). A novel strategy of integrated microarray analysis identifies CENPA, CDK1 and CDC20 as a cluster of diagnostic biomarkers in lung adenocarcinoma. *Cancer Letters*.

[25] Yue C., Ma H., Zhou Y. (2019). Identification of prognostic gene signature associated with microenvironment of lung adenocarcinoma. *PeerJ*.

[26] Wang Z., Embaye K. S., Yang Q. (2021). Establishment and validation of a prognostic signature for lung adenocarcinoma based on metabolism-related genes. *Cancer Cell International*.

[27] Al-Dherasi A., Huang Q. T., Liao Y. (2021). A seven-gene prognostic signature predicts overall survival of patients with lung adenocarcinoma (LUAD). *Cancer Cell International*.

[28] He L., Chen J., Xu F., Li J., Li J. (2020). Prognostic implication of a metabolism-associated gene signature in lung adenocarcinoma. *Molecular Therapy - Oncolytics*.

[29] Jin J., Liu C., Yu S. (2021). A novel ferroptosis-related gene signature for prognostic prediction of patients with lung adenocarcinoma. *Aging*.

[30] Hardavella G., George R., Sethi T. (2016). Lung cancer stem cells-characteristics, phenotype. *Translational Lung Cancer Research*.

[31] Miyoshi N., Mizushima T., Doki Y., Mori M. (2019). Cancer stem cells in relation to treatment. *Japanese Journal of Clinical Oncology*.

[32] Shibata M., Hoque M. O. (2019). Targeting Cancer Stem Cells: A Strategy for Effective Eradication of Cancer. *Cancers*.

[33] Suo H. D., Tao Z., Zhang L. (2020). Coexpression network analysis of genes related to the characteristics of tumor stemness in triple-negative breast cancer. *BioMed Research International*.

[34] Guo R., Chu A., Gong Y. (2020). Identification of cancer stem cell-related biomarkers in intestinal-type and diffuse-type gastric cancer by stemness index and weighted correlation network analysis. *Journal of Translational Medicine*.

[35] Bai K. H., He S. Y., Shu L. L. (2020). Identification of cancer stem cell characteristics in liver hepatocellular carcinoma by WGCNA analysis of transcriptome stemness index. *Cancer Medicine*.

[36] Liao Y., Xiao H., Cheng M., Fan X. (2020). Bioinformatics analysis reveals biomarkers with cancer stem cell characteristics in lung squamous cell carcinoma. *Frontiers in Genetics*.

[37] Testa U., Castelli G., Pelosi E. (2018). Lung cancers: molecular characterization, clonal heterogeneity and evolution, and cancer stem cells. *Cancers*.

[38] Imielinski M., Berger A. H., Hammerman P. S. (2012). Mapping the hallmarks of lung adenocarcinoma with massively parallel sequencing. *Cell*.

[39] Wang Z., Wang C., Lin S., Yu X. (2021). Effect of TTN mutations on immune microenvironment and efficacy of immunotherapy in lung adenocarcinoma patients. *Frontiers in Oncology*.

[40] Liu P., Morrison C., Wang L. (2012). Identification of somatic mutations in non-small cell lung carcinomas using whole-exome sequencing. *Carcinogenesis*.

[41] Wang C., Liang H., Lin C. (2019). Molecular subtyping and prognostic assessment based on tumor mutation burden in patients with lung adenocarcinomas. *International Journal of Molecular Sciences*.

[42] Lan S., Li H., Liu Y. (2019). Somatic mutation of LRP1B is associated with tumor mutational burden in patients with lung cancer. *Lung Cancer*.

[43] Muller L., Tunger A., Plesca I. (2020). Bidirectional crosstalk between cancer stem cells and immune cell subsets. *Frontiers in Immunology*.

[44] Lopez-Lazaro M. (2018). The stem cell division theory of cancer. *Critical Reviews in Oncology/Hematology*.

[45] Wu Y., Liu L., Shen X., Liu W., Ma R. (2021). Plakophilin-2 promotes lung adenocarcinoma development via enhancing focal adhesion and epithelial-mesenchymal transition. *Cancer Management and Research*.

[46] Liu W., Jiang K., Wang J., Mei T., Zhao M., Huang D. (2021). Upregulation of GNPNAT1 predicts poor prognosis and correlates with immune infiltration in lung adenocarcinoma. *Frontiers in Molecular Biosciences*.

[47] Zheng X., Li Y., Ma C. (2020). Independent prognostic potential of GNPNAT1 in lung adenocarcinoma. *BioMed Research International*.

[48] Zhao M., Chen Z., Zheng Y. (2020). Identification of cancer stem cell-related biomarkers in lung adenocarcinoma by stemness index and weighted correlation network analysis. *Journal of Cancer Research and Clinical Oncology*.

[49] Yao X., Ireland S. K., Pham T. (2014). TLE1 promotes EMT in A549 lung cancer cells through suppression of E-cadherin. *Biochemical and Biophysical Research Communications*.

[50] Borrelli A., Schiattarella A., Mancini R. (2009). A recombinant MnSOD is radioprotective for normal cells and radiosensitizing for tumor cells. *Free Radical Biology and Medicine*.

